# *Deqi* Sensation to Predict Acupuncture Effect on Functional Dyspepsia: A Machine Learning Study

**DOI:** 10.1155/2022/4824575

**Published:** 2022-09-14

**Authors:** Li Chen, Tao Yin, Zhaoxuan He, Yuan Chen, Ruirui Sun, Jin Lu, Peihong Ma, Fang Zeng

**Affiliations:** ^1^Acupuncture and Tuina School, The 3rd Teaching Hospital, Chengdu University of Traditional Chinese Medicine, Chengdu 610075, China; ^2^Acupuncture-Brain Research Center, Chengdu University of Traditional Chinese Medicine, Chengdu 610075, China; ^3^Key Laboratory of Sichuan Province for Acupuncture and Chronobiology, Chengdu 610075, China; ^4^International Education School, Chengdu University of Traditional Chinese Medicine Chengdu, Chengdu 610075, China; ^5^School of Acupuncture-Moxibustion and Tuina, Beijing University of Chinese Medicine, Beijing 100029, China

## Abstract

**Objectives:**

The aim of the study was to predict the effect of acupuncture for treating functional dyspepsia (FD) using the support vector machine (SVM) techniques based on initial *deqi* sensations of patients.

**Methods:**

This retrospective study involved 90 FD patients who had received four weeks of acupuncture treatment. The support vector classification model was used to distinguish higher responders (patients with Symptom Index of Dyspepsia improvement score ≥ 2) from lower responders (patients with Symptom Index of Dyspepsia improvement score < 2). A support vector regression model was used to predict the change in the Symptom Index of Dyspepsia at the end of acupuncture treatment. *Deqi* sensations of patients in the first acupuncture treatment of a 20-session acupuncture intervention were defined as features and used to train models. Models were validated by 10-fold cross-validation and evaluated by accuracy, specificity, sensitivity, the area under the receive-operating curve, the coefficient of determination (*R*^2^), and the mean squared error.

**Results:**

The two models could predict the efficacy of acupuncture successfully. These models had an accuracy of 0.84 in predicting acupuncture response, and an *R*^2^ of 0.16 in the prediction of symptom improvements, respectively. The presence or absence of *deqi* sensation, the duration of *deqi* sensation, distention, and pain were finally selected as significant predicting features.

**Conclusion:**

Based on the SVM algorithms and *deqi* sensation, the current study successfully predicted the acupuncture response as well as clinical symptom improvement in FD patients at the end of treatment. Our prediction models are expected to promote the clinical efficacy of acupuncture treatment for FD, reduce medical expenditures, and optimize the allocation of medical resources.

## 1. Introduction

Functional dyspepsia (FD) is defined as chronic discomfort or pain originating from the epigastric region without underlying organic lesions [1]. FD has a high prevalence ranging from 8% to 12% worldwide [2], which is associated with poor psychophysiological health and quality of life (QoL) of patients [3] and a high economic burden on individuals and communities [4]. Acupuncture has long been recognized as a potentially effective complementary and alternative medicine (CAM) therapy for the treatment of functional gastric disorders. Several high-quality clinical trials have validated the therapeutic efficacy of acupuncture in treating FD [5–8]. For instance, our previous studies demonstrated that acupuncture relieved FD symptoms and improved the QoL of FD patients [6, 7]. In addition, the study found that the efficacy of acupuncture in improving QoL was more pronounced than itopride, a recommended medicine for FD [6]. However, as a typical individualized therapy, acupuncture is not effective for all patients with FD because of the varying responses to acupuncture stimulation [9, 10]. Furthermore, we found that acupuncture with *deqi* sensations relieved the symptoms of FD better than acupuncture without *deqi* sensations [11]. The *deqi* sensation, also known as the needling sensation, comprises unique sensations including but not limited to soreness, numbness, heaviness, distension, warmth, coldness, and pain experienced by the patients around the acupoints during acupuncture manipulation [12, 13]. The *deqi* sensation is key to the therapeutic effect of acupuncture, which has been highlighted in traditional Chinese acupuncture theory (e.g., “*Deqi* is the precondition of acupuncture stimulation to obtain a therapeutic effect”) and has been proven in clinical practices [14–20]. These findings suggested the significant impacts of *deqi* sensations on the efficacy of acupuncture in treating FD and raised the question of whether the acupuncture effect could be predicted based on patients' *deqi* sensations.

Recently, machine learning (ML) techniques have been widely used for the prediction of clinical efficacy and decision-making in medicine [21, 22] and have been regarded as powerful tools for predictive, preventive, and personalized medicine (PPPM/3PM) [23]. The PPPM/3PM is an advanced philosophy in healthcare and disease care sectors used to predict individual predisposition to a disease, provide targeted preventive measures, and develop personalized treatment strategies tailored to the individual [24–26]. Among ML algorithms, the support vector machine (SVM) is most used in efficacy prediction because of its outstanding performance and strong generalization [27, 28]. Several studies have reported that SVM based on baseline functional neuroimaging features can effectually distinguish patients from healthy subjects and predict acupuncture efficacy [29–32]. However, because of the difficulties in neuroimaging data acquisition and processing, the translational potential of these prediction models is substantially limited. Therefore, it is of great practical value to explore a more accessible approach to predicting acupuncture efficacy in treating FD.

In the framework of PPPM/3PM, this study developed two prediction models based on the SVM algorithm and the patient's initial *deqi* sensations, with an aim of predicting (1) treatment response and (2) clinical symptom improvement in FD patients at the end of treatment. This study is expected to provide a valuable reference for the application of PPPM/3PM in CAM, help doctors in identifying patients appropriate for acupuncture treatment, and ultimately develop personalized treatment tailored to the individual.

## 2. Materials and Methods

### 2.1. Study Design

This study was a priori planned secondary analysis involving 90 participants selected from the Affiliated Hospital of Chengdu University of Traditional Chinese Medicine (CDUTCM) and the campus of CDUTCM from January 2016 to May 2018. The entire study period consisted of six weeks, including a two-week run-in period and a four-week treatment period. The study was performed according to the Declaration of Helsinki and was registered in the Chinese Clinical Trial Registry (registration number: ChiCTR-IOR-15006523). Ethics approval was granted by the Institutional Review Board of Affiliated Hospital of CDUTCM (approval number: 2015KL-002).

### 2.2. Participants

The patients were included if they (1) were 18 to 45 years old, (2) met Rome III criteria for FD, (3) did not attend any other clinic trials, and (4) provided written informed consent.

On the other hand, patients were excluded if they (1) had organic gastrointestinal disorders such as esophagitis, gastric atrophy, or erosive gastroduodenal lesions on endoscopy, (2) had infection overlapping with the acupuncture sites, (3) received acupuncture treatment three months before baseline, (4) were taking medications affecting gastrointestinal motility such as nonsteroidal anti-inflammatory drugs and selective serotonin reuptake inhibitors two weeks before baseline, (5) were pregnant, lactating or had childbearing potential but not using adequate contraception, or (6) had severe mental disorders such as anxiety and depression.

### 2.3. Randomized Allocation and Blinding

Eligible participants were randomly assigned to two groups (Shu-Mu acupoints group and He-Mu acupoints group) with a 1 : 1 ratio. The randomization sequence was generated using a central computer system, which ensured that they were well concealed throughout the trial. Because of the nature of acupuncture, blinding participants and investigators to the group assignment is difficult. To minimize bias, outcomes were measured at baseline and the end of acupuncture treatment after randomization by the same independent assessors who were blinded to the allocation system.

### 2.4. Acupuncture Interventions

Acupoints bilateral *Weishu* (BL21) and *Zhongwan* (CV12) were selected in the Shu-Mu acupoints group whereas bilateral *Zusanli* (ST36) and CV12 were selected in the He-Mu acupoints group (Figure 1). All patients received 20 sessions of manual acupuncture treatment lasting 30 minutes each over four weeks (5 sessions per week), and each acupuncture session lasted 30 minutes. The *deqi* sensations were required as much as possible in each acupoints. Two licensed acupuncturists with over three years of clinical experience performed acupuncture interventions.

### 2.5. Outcome Measurement

The Symptom Index of Dyspepsia (SID) was utilized to measure dyspepsia symptoms in FD patients at baseline and at the end of acupuncture treatment. SID is a four-rate scale scored in the 0–4 range for each dyspepsia symptom (postprandial distension, early satiety, epigastric pain, and epigastric burning) [6]. Higher scores indicate more severe symptoms. FD patients with SID improvement scores ≥ 2 were regarded as higher responders, whereas FD patients with SID improvement scores < 2 were grouped as lower-responders.

### 2.6. *Deqi* Sensations Evaluations

A Chinese version of the Massachusetts General Hospital Acupuncture Sensation Scale (C-MASS) [33] was used to record the patients' initial sensations of acupuncture. The 10-point Visual Analog Scale was used to assess the five types of *deqi* sensations, namely, soreness, numbness, distention, heaviness, and pain [34]. To adequately describe *deqi* sensation, the presence or absence of *deqi* sensations (1 means with *deqi* sensations, 0 means without *deqi* sensations), the total score of *deqi* sensations (total score of five main *deqi* sensations score), and the duration of *deqi* sensations (ranges from 1 to 4, and the larger the number, the longer the duration) were recorded.

### 2.7. Statistical Analysis

#### 2.7.1. Demographic and Clinical Characteristics

The SPSS 22.0 statistics software (IBM SPSS Statistics, IBM Corp, Somers, New York) was used to analyze demographic and clinical features. Continuous data were expressed as mean and standard deviation (mean ± SD), and the Shapiro–Wilk test was used to verify whether the data were normally distributed. Between-group comparisons were performed using the two independent sample *t*-tests or Mann–Whitney *U* tests for normally distributed data and non-normal data, and within-group comparisons were performed using the linear mixed model. The chi-squared test (*χ*2) test was used for categorical variables. The significance level was set at *P* < 0.01 (two-tailed).

### 2.8. Support Vector Machine Analysis

#### 2.8.1. Classification of Acupuncture Responders

Higher responders were labeled “1,” whereas the lower responders were labeled “−1.” The patients' initial *deqi* sensations included the presence or absence of *deqi* sensations, the type of *deqi* sensations (soreness, numbness, distention, heaviness, and pain), the total score of *deqi* sensations, and the duration of *deqi* sensations. These eight parameters of *deqi* sensations were selected as input features. Afterward, a linear kernel support vector classification (SVC) with default parameters was employed to build a classifier between higher responders and lower responders based on the LIBSVM toolbox [35] in Matlab 2017b. 10-fold cross-validation was used to evaluate the performance of this classification model, with accuracy, specificity, sensitivity, and the area under the receive-operating curve (AUC) as evaluation indicators. In the 10-fold cross-validation, the sample was divided into ten equally sized folds. Nine folds were used to train the model, whereas the remaining one was used to test the performance of the model. The significance of the analysis results was measured using permutation testing (permutation times = 1,000). The classification process was performed in 1000 iterations to reduce errors caused by the random division of samples in 10-fold cross-validation. Lastly, the accuracy, specificity, sensitivity, and AUC were described as mean ± SD of 1000 iterations.

#### 2.8.2. Prediction of Symptom Improvement

This study further performed a prediction analysis of symptom improvement in FD patients. The linear kernel support vector regression (SVR) algorithm based on eight parameters of *deqi* sensations was used to construct a prediction model to predict symptom improvement (changes in SID scores after treatment) in FD patients. Similar to the classification analysis of acupuncture responders, the 10-fold cross-validation was used to evaluate the prediction model. The performance of this model was assessed using the coefficient of determination (*R*^2^) and the mean squared error (MSE). The *R*^2^ was defined as the square of the correlation between the actual and predicted treatment response. The MSE was defined as the expectation of the square of the difference between the actual and predicted treatment response. The permutation tests (permutation times = 1,000) were used to estimate the significance of *R*^2^ and MSE. The prediction procedure was also repeated 1000 times to reduce the error generated by the random division of the samples during the 10-fold cross-validation. Finally, *R*^2^ and MSE were described as mean ± SD of 1000 iterations.

#### 2.8.3. Calculation of Feature Weights

The weight of the feature reflects the magnitude of each feature's contribution to determining the support vector classification hyperplane. The larger the value of a feature weight, the greater its contribution to the classification results. In this study, the weight of features in the 10-fold cross-validation was calculated. Similar to the model performance evaluation, the weight of features was determined using an average of 1000 iterations.

## 3. Results

According to the SID improvement, 55 FD patients were grouped as the higher responders, whereas 35 FD patients were grouped as the lower-responders. The study flowchart was displayed in Figure 2.

### 3.1. Demographic and Clinical Characteristics

There were no significant differences in the age, gender, body mass index (BMI), and duration of disease between the higher responders and lower responders groups (all *p* > 0.05; Table 1). Except for the pain, the score of the other four types of *deqi* sensations, duration of *deqi* sensations, and total score of *deqi* sensations in the higher responders group were higher than those in the lower-responders group (all *p* < 0.05; Table 1). The baseline SID score and the SID improvement score of higher responders were markedly greater than those of lower responders (all *p* < 0.01; Table 1).

### 3.2. Pattern Classification

The overall linear kernel SVC model achieved an accuracy of 0.84 ± 1.72, AUC of 0.90 ± 0.01, the sensitivity of 0.88 ± 0.02, and specificity of 0.79 ± 0.03 in classifying acupuncture responders (Figures 3(a) and 3(e)). Results of the permutation test showed that the accuracy and AUC were both significant (*p*_accuracy < 0.001, *p*_AUC < 0.001) (Figures 3(f) and 3(g)).

### 3.3. Prediction of Acupuncture Efficacy

The prediction model obtained a *R*^2^ of 0.16 ± 0.02 between actual and predicted symptom improvement and an MSE of 1.64 ± 0.07 for acupuncture treatment (Figures 4(a) and 4(b)). The correlation between the actual and predicted improvement of SID was displayed in Figures 3(c) and 3(e). Results of the permutation test showed that the MSE and *R*^2^ were both significant (*p*_MSE = 0.016, *p*_*R*^2^ = 0.022) (Figures 4(f) and 4(g)).

### 3.4. Weight of Predicting Features

As shown in Figure 5(a), the distention (weight = 0.851) and pain (weight = 0.60) were the most weighted features for the prediction of acupuncture response. As shown in Figure 5(b), the presence or absence of *deqi* sensation (weight = 0.288), the duration of *deqi* sensation (weight = 0.242), and distention (weight = 0.202) were the most weighted features for the prediction of SID improvement score.

## 4. Discussion

Combining the SVM algorithms and initial *deqi* sensation, the current study successfully predicted the acupuncture response as well as clinical symptom improvement in FD patients at the end of treatment. These findings provided a reliable reference for applying PPPM/3PM in CAM and demonstrated that initial *deqi* sensations of patients could be valuable predictors of acupuncture efficacy.

### 4.1. SVM Is a Reliable Approach to Predicting Acupuncture Efficacy

Personalized diagnosis and clinical efficacy prediction based on ML technologies have been researched hotspots in recent years because studies have shown that treatment personalization is the future of medicine [36–41]. As a supervised ML technique, SVM is a maximum fringe hyperplane that lies in some space to separate the two groups by minimizing the empirical classification error in training data to achieve a higher degree of accuracy for unseen data [42]. In recent years, SVM has become increasingly popular in the classification and acupuncture efficacy prediction research [9, 29–31, 43]. Additionally, studies show that SVM performs better than conventional generalized linear models in classifying and predicting intricate data. For example, Yin et al. compared the performance of several common ML algorithms (e.g., decision tree, logistic regression, K-nearest neighbor, and boosted tree) in predicting acupuncture efficacy and found that the prediction models constructed based on the SVM algorithm had better performance than others [44]. This study also demonstrated the feasibility of using SVM to predict acupuncture's effectiveness, highlighting the reliability and value of SVM. Whether based on objective neuroimaging characteristics or subjective perceptions data, the SVM exhibits outstanding performance in prediction analysis.

### 4.2. Prediction Models Developed with Deqi Sensation Have Better Translational Potential

Recent studies have applied the SVM algorithm and novel biomarkers, such as functional neuroimaging data, to predict the acupuncture effect, yielding encouraging results. For example, our previous study found that SVM based on the whole-brain functional network at baseline could successfully forecast the efficacy of acupuncture on FD [32]. Moreover, SVM combined with cerebral activity pattern at baseline was found to effectively predict relief of monthly migraine days after a 4-week acupuncture treatment [29]. However, neuroimaging data, especially high-field magnetic resonance data, are still difficult to acquire and process in primary healthcare, limiting the clinical applications of these novel prediction models and biomarkers. In contrast, the prediction models constructed with features collected in routine practice may have greater translational potential. Although the *deqi* sensation is not an objective indicator, it can be easily determined from patient responses. More importantly, the *deqi* sensation is a highly individualized clinical indicator, which may be perceived differently by patients perceiving the same acupuncture stimulation. The development of an efficacy prediction model constructed with the input feature of *deqi* sensations will potentially promote personalized medicine. Therefore, the prediction models based on the *deqi* sensation developed in this study have better translational potential.

### 4.3. The Presence or Absence of Deqi Sensation, Duration of Deqi Sensation, Distention, and Pain Are Useful Features for Precise Predictions

The *deqi* sensation is considered an important parameter in achieving the therapeutic effects of acupuncture treatment [45, 46]. For instance, acupuncture with *deqi* sensations contributed to higher response and elimination rates of postprandial fullness, upper abdominal bloating, and early satiation in patients with FD than sham acupuncture without *deqi* sensations [5, 11]. Therefore, the presence or absence of *deqi* sensation can be used as a predictor of FD symptoms. Many Chinese medical texts state that the duration of the *deqi* sensation also influences the acupuncture effect. For example, Chinese acupuncture therapy involves repeated needling manipulations over the needle retention period to extend the duration of the *deqi* sensations as long as possible [11]. This study found that the duration of *deqi* sensation in the higher-responders' group was longer than in the lower-responders' group. As a result, the duration of the *deqi* sensation can be considered another key predictor of acupuncture efficacy for FD. As the type of *deqi* sensation reported most frequently by patients receiving acupuncture treatment [10, 47], distention was proven to be associated with the therapeutic efficacy of acupuncture. Studies have shown that distention was related to the improvement of facial nerve function in patients with Bell's palsy, and the greater intensity of distension could predict a better acupuncture outcome [48]. In this study, the intensity of distention in the higher-responders' group was stronger than that in the lower-responders' group. Results from this study suggested that the intensity of distention can be a reasonable predictor to identify the responders of acupuncture treatment for FD. Lastly, pain was also found to be predictive of the efficacy of acupuncture treatment for FD. However, there was no significant difference in pain intensity between the two groups. It was speculated that the mild pain was due to the penetration of the needle into the skin and muscles. However, whether this pain is related to the efficacy of acupuncture remains unclear. Besides, SVM has major drawbacks known as the black-box effects, which imply the opacity of the data processing and the subsequent difficulty in explaining the results. Further studies are required to elucidate the contribution of pain to the prediction of the efficacy of acupuncture for FD.

## 5. Conclusion

In summary, this study constructed SVM prediction models based on the initial *deqi* sensations, which successfully predicted the acupuncture response and symptom improvement in FD patients at the end of treatment. As a preliminary study, it has some limitations including smaller sample size and the lack of objective outcome measurement for FD treatment. However, our results highlighted the value of integrating ML techniques and *deqi* sensation to predict the efficacy of acupuncture and provided a novel approach to facilitate the application of PPPM/3PM in CAM. These prediction models are expected to promote the clinical efficacy of acupuncture treatment for FD, reduce medical expenditures, and optimize the allocation of medical resources.

## Figures and Tables

**Figure 1:** The location of acupoints. *Weishu* (BL21): on the back, 1.5 cun lateral to the lower border of the spinous process of the 12th thoracic vertebra; *Zusanli* (ST36): on the anterior lateral side of the shank, 3 cun below *Dubi* (ST35), one horizontally placed finger distance lateral to the anterior border of the tibia; *Zhongwan* (CV12): on the anterior median line of the upper abdomen, 4 cun above the navel.

**Figure 2:** Study flowchart. FD, functional dyspepsia; SID, symptom index of dyspepsia; SVC, support vector classification; SVR, support vector regression.

**Figure 3:** Results of classification analyses. (a–d) The frequency distribution of accuracy, specificity, sensitivity, and AUC after 1000 iterations in the SVC model. (e) The ROC curves of the SVC model for 1000 iterations, with each line representing one iteration. (f) Real AUC was significantly higher than pseudo-AUC generated by permutation testing (*p* < 0.001). (g) Real accuracy was significantly higher than pseudo accuracy generated by Permutation testing (*p* < 0.001). AUC, area under the receiver-operating characteristic curve; ROC, receiver-operating characteristic. SVC, support vector classification.

**Figure 4:** Results of prediction analyses. (a) The frequency distribution of MSE after 1000 iterations in the SVR model. (b) The frequency distribution of *R*^2^ after 1000 iterations in the SVR model. (c and e) The correlation scatterplots between the actual values and predicted values, the scatterplots for the best predictive performance (Max), the average predictive performance (Mean), and the worst predictive performance (Min) in the 1000 repetitions were plotted, respectively. (f) Real MSE was significantly lower than pseudo-MSE generated by Permutation testing (*p*=0.016). (g) Real *R*^2^ was significantly higher than pseudo *R*^2^ generated by Permutation testing (*p*=0.022). SVR, support vector regression; MSE, mean squared error; *R*^2^, coefficient of determination.

**Figure 5:** Weight of features. (a) The weight of features in the SVC model. (b) The weight of features in the SVR model. SVC, support vector classification; SVR, support vector regression.

**Table 1:** Demographic and clinical characteristics of the participants.

Item	Higher responders (*n* = 55)	Lower responders (*n* = 35)	*Z*/*χ*^2^	*p* value
Age (years)	22.35 ± 2.46	22.23 ± 2.90	−0.648	0.517
Gender (female), *n* (%)	49 (89.1)	26 (74.3)	3.376	0.066
BMI (kg/m^2^)	19.92 ± 2.83	20.05 ± 1.80	−0.269	0.788
Duration (months)	45.87 ± 27.74	41.29 ± 39.68	−1.321	0.186
The duration of *deqi* sensations (minutes)	22.91 ± 7.24	13.86 ± 8.46	−4.626	< 0.001
The total score of *deqi* sensations	15.14 ± 8.97	6.60 ± 4.13	−5.011	< 0.001
Soreness	1.96 ± 2.13	0.86 ± 1.24	−2.391	0.017
Numbness	2.13 ± 2.40	0.51 ± 0.95	−3.764	< 0.001
Heaviness	2.40 ± 2.48	0.89 ± 1.23	−2.718	0.007
Distention	5.65 ± 1.63	2.43 ± 1.61	−6.767	< 0.001
Pain	1.93 ± 2.17	1.23 ± 1.50	−1.391	0.164
Pre-treatment SID	4.29 ± 1.36	2.63 ± 0.88	−5.574	< 0.001
Post-treatment SID	1.45 ± 0.94	1.86 ± 0.91	−1.956	0.050
SID change sores	2.84 ± 1.12	0.77 ± 0.49	−8.252	< 0.001

Results are presented as mean ± SD or number (percentage). BMI, body mass index; SID, symptom index of dyspepsia.

## Data Availability

The datasets and codes are available upon reasonable request via e-mail to the corresponding author (zengfang@cdutcm.edu.cn).

## References

[1] Stanghellini V., Chan F. K., Hasler W. L. (2016). Gastroduodenal disorders. *Gastroenterology*.

[2] Aziz I., Palsson O. S., Törnblom H., Sperber A. D., Whitehead W. E., Simren M. (2018). Epidemiology, clinical characteristics, and associations for symptom-based Rome IV functional dyspepsia in adults in the USA, Canada, and the UK: a cross-sectional population-based study. *The Lancet Gastroenterology & Hepatology*.

[3] Ford A. C., Mahadeva S., Carbone M. F., Lacy B. E., Talley N. J. (2020). Functional dyspepsia. *The Lancet*.

[4] Brook R. A., Kleinman N. L., Choung R. S., Melkonian A. K., Smeeding J. E., Talley N. J. (2010). Functional dyspepsia impacts absenteeism and direct and indirect costs. *Clinical Gastroenterology and Hepatology*.

[5] Yang J. W., Wang L. Q., Zou X. (2020). Effect of acupuncture for postprandial distress syndrome: a randomized clinical trial. *Annals of Internal Medicine*.

[6] Ma T. T., Yu S. Y., Li Y. (2012). Randomised clinical trial: an assessment of acupuncture on specific meridian or specific acupoint vs. sham acupuncture for treating functional dyspepsia. *Alimentary Pharmacology and Therapeutics*.

[7] Zheng H., Xu J., Sun X. (2018). Electroacupuncture for patients with refractory functional dyspepsia: a randomized controlled trial. *Neuro-Gastroenterology and Motility*.

[8] Zeng F., Qin W., Ma T. (2012). Influence of acupuncture treatment on cerebral activity in functional dyspepsia patients and its relationship with efficacy. *American Journal of Gastroenterology*.

[9] Yang X. J., Liu L., Xu Z. L. (2020). Baseline brain gray matter volume as a predictor of acupuncture outcome in treating migraine. *Frontiers in Neurology*.

[10] Mao J. J., Farrar J. T., Armstrong K., Donahue A., Ngo J., Bowman M. A. (2007). De qi: Chinese acupuncture patients’ experiences and beliefs regarding acupuncture needling sensation-an exploratory survey. *Acupuncture in Medicine*.

[11] Sun R., He Z., Ma P. (2021). The participation of basolateral amygdala in the efficacy of acupuncture with deqi treating for functional dyspepsia. *Brain Imaging and Behavior*.

[12] Kong J., Gollub R., Huang T. (2007). Acupuncture de qi, from qualitative history to quantitative measurement. *Journal of Alternative & Complementary Medicine*.

[13] Hui K. K., Sporko T. N., Vangel M. G., Li M., Fang J., Lao L. (2011). Perception of deqi by Chinese and American acupuncturists: a pilot survey. *Chinese Medicine*.

[14] Spaeth R. B., Camhi S., Hashmi J. A. (2013). A longitudinal study of the reliability of acupuncture deqi sensations in knee osteoarthritis. *Evidence-Based Complementary and Alternative Medicine*.

[15] Shi G. X., Li Q. Q., Liu C. Z. (2014). Effect of acupuncture on deqi traits and pain intensity in primary dysmenorrhea: analysis of data from a larger randomized controlled trial. *BMC Complementary and Alternative Medicine*.

[16] Zhao M. Y., Zhang P., Li J. (2017). Influence of de qi on the immediate analgesic effect of SP6 acupuncture in patients with primary dysmenorrhoea and cold and dampness stagnation: a multicentre randomised controlled trial. *Acupuncture in Medicine*.

[17] Li H., Liu H., Liu C. (2014). Effect of “deqi” during the study of needling “Wang’s Jiaji” acupoints treating spasticity after stroke. *Evidence-Based Complementary and Alternative Medicine*.

[18] Yin X., Gou M., Xu J. (2017). Efficacy and safety of acupuncture treatment on primary insomnia: a randomized controlled trial. *Sleep Medicine*.

[19] Xu S. B., Huang B., Zhang C. Y. (2013). Effectiveness of strengthened stimulation during acupuncture for the treatment of bell palsy: a randomized controlled trial. *Canadian Medical Association Journal*.

[20] Witt C., Brinkhaus B., Jena S. (2005). Acupuncture in patients with osteoarthritis of the knee: a randomised trial. *The Lancet*.

[21] Waljee A. K., Higgins P. D. R. (2010). Machine learning in medicine: a primer for physicians. *American Journal of Gastroenterology*.

[22] Pappada S. M. (2021). Machine learning in medicine: it has arrived, let’s embrace it. *Journal of Cardiac Surgery*.

[23] Barrett M., Boyne J., Brandts J. (2019). Artificial intelligence supported patient self-care in chronic heart failure: a paradigm shift from reactive to predictive, preventive and personalised care. *The EPMA Journal*.

[24] Golubnitschaja O., Kinkorova J., Costigliola V. (2014). Predictive, preventive and personalised medicine as the hardcore of “horizon 2020”: EPMA position paper. *The EPMA Journal*.

[25] Golubnitschaja O., Baban B., Boniolo G. (2016). Medicine in the early twenty-first century: paradigm and anticipation-EPMA position paper 2016. *The EPMA Journal*.

[26] Islam F., Khadija J. F., Harun-Or-Rashid M. (2022). Bioactive compounds and their derivatives: an insight into prospective phytotherapeutic approach against alzheimer’s disease. *Oxidative Medicine and Cellular Longevity*.

[27] Vidyasagar M. (2015). Identifying predictive features in drug response using machine learning: opportunities and challenges. *Annual Review of Pharmacology and Toxicology*.

[28] Wu Z., Zhu M., Kang Y. (2021). Do we need different machine learning algorithms for QSAR modeling? A comprehensive assessment of 16 machine learning algorithms on 14 QSAR data sets. *Briefings in Bioinformatics*.

[29] Yin T., Sun G., Tian Z. (2020). The spontaneous activity pattern of the middle occipital gyrus predicts the clinical efficacy of acupuncture treatment for migraine without aura. *Frontiers in Neurology*.

[30] Tu Y., Ortiz A., Gollub R. L. (2019). Multivariate resting-state functional connectivity predicts responses to real and sham acupuncture treatment in chronic low back pain. *NeuroImage Clinical*.

[31] Tu Y., Zeng F., Lan L. (2020). An fMRI-based neural marker for migraine without aura. *Neurology*.

[32] Yin T., Sun R., He Z., Ma P. H, Zeng F. (2020). Clinical effects of acupuncture treatment in functional dyspepsia based on resting-state functional brain network. *China Journal of Traditional Chinese Medicine and Pharmacy*.

[33] Yu D. T. W., Jones A. Y. M., Pang M. Y. C. (2012). Development and validation of the Chinese version of the Massachusetts general hospital acupuncture sensation scale: an exploratory and methodological study. *Acupuncture in Medicine*.

[34] Ren Y. L., Guo T. P., Du H. B. (2015). A survey of the practice and perspectives of Chinese acupuncturists on deqi. *Evidence-Based Complementary and Alternative Medicine*.

[35] Chang C. C., Lin C. J. (2011). LIBSVM: a library for support vector machines. *ACM Transactions on Intelligent Systems and Technology*.

[36] Zeevi D., Korem T., Zmora N. (2015). Personalized nutrition by prediction of glycemic responses. *Cell*.

[37] Montazeri M., Montazeri M., Montazeri M., Beigzadeh A. (2016). Machine learning models in breast cancer survival prediction. *Technology and Health Care*.

[38] de Jong J., Cutcutache I., Page M. (2021). Towards realizing the vision of precision medicine: AI based prediction of clinical drug response. *Brain*.

[39] Oikonomou E. K., Williams M. C., Kotanidis C. P. (2019). A novel machine learning-derived radiotranscriptomic signature of perivascular fat improves cardiac risk prediction using coronary CT angiography. *European Heart Journal*.

[40] Motwani M., Dey D., Berman D. S. (2017). Machine learning for prediction of all-cause mortality in patients with suspected coronary artery disease: a 5-year multicentre prospective registry analysis. *European Heart Journal*.

[41] Trebeschi S., Drago S. G., Birkbak N. J. (2019). Predicting response to cancer immunotherapy using noninvasive radiomic biomarkers. *Annals of Oncology*.

[42] Nayak J., Naik B., Behera H. S. (2015). A comprehensive survey on support vector machine in data mining tasks: applications & challenges. *International Journal of Database Theory and Application*.

[43] Yu S., Xie M., Liu S. (2020). Resting-state functional connectivity patterns predict acupuncture treatment response in primary dysmenorrhea. *Frontiers in Neuroscience*.

[44] Yin T., Zheng H., Ma T. (2022). Predicting acupuncture efficacy for functional dyspepsia based on routine clinical features: a machine learning study in the framework of predictive, preventive, and personalized medicine. *The EPMA Journal*.

[45] Zhou W., Benharash P. (2014). Significance of “Deqi” response in acupuncture treatment: myth or reality. *Journal of Acupuncture and Meridian Studies*.

[46] Yuan H. W., Ma L. X., Zhang P. (2013). An exploratory survey of deqi sensation from the views and experiences of Chinese patients and acupuncturists. *Evidence-Based Complementary and Alternative Medicine*.

[47] Lu F. Y., Gao J. H., Wang Y. Y. (2021). Effects of three needling manipulations of Zusanli (ST 36) on deqi sensations and surface myoelectricity in healthy participants. *Chinese Journal of Integrative Medicine*.

[48] Zhang C. Y., Xu S. B., Huang B. (2016). Needle sensation and personality factors influence therapeutic effect of acupuncture for treating bell’s palsy: a secondary analysis of a multicenter randomized controlled trial. *Chinese Medical Journal*.

